RETRACTED

# The efficacy and safety of neubotulinumtoxinA for the treatment of forehead horizontal lines in Asians – A clinical, prospective, interventional, split‐face study

**DOI:** 10.1111/srt.13644

**Published:** 2024-03-27

**Authors:** Jessica Jane Sy, Raymond Wu, Jovian Wan, Soo‐Bin Kim, Kyu‐Ho Yi

**Affiliations:** ^1^ Asia‐Pacific Aesthetic Academy Seoul Hong Kong; ^2^ Division in Anatomy and Developmental Biology, Department of Oral Biology Human Identification Research Institute, BK21 FOUR Project, Yonsei University College of Dentistry, 50–1 Yonsei‐ro, Seodaemun‐gu Seoul South Korea; ^3^ Maylin Clinic (Apgujeong) Seoul South Korea

**Keywords:** botulinum toxin, horizontal forehead lines, neuromodulators, split‐face study

## Abstract

**Background:**

Botulinum toxin injections are widely sought after in the field of medical aesthetics, offering consumers a variety of brand choices. Two commonly available botulinum toxin products, onabotulinumtoxinA and neubotulinumtoxinA, are featured in numerous clinics, leading many to question whether there are discernible differences in results, given their varying price ranges.

**Objective:**

To evaluate the efficacy and safety of neubotulinumtoxinA for the treatment of forehead horizontal lines.

**Methods:**

A 12‐week prospective, single‐centre, interventional split‐face study was conducted, including 30 subjects. These enrolled subjects received a single treatment session, with neubotulinumtoxinA applied to the left side of the forehead and onabotulinumtoxinA to the right side. A superficial injection was performed in all individuals, where the product was injected subdermally in the frontalis muscle. Evaluation was conducted at baseline, 7 days, 14, days and 4, 8, and 12 weeks after treatment, both when the eyebrows were at maximum lift and in a resting position. Treatment efficacy was assessed by two physicians and self‐assessed by the patients, using the Fitzpatrick Wrinkle Classification system. Adverse events were documented to evaluate safety.

**Results:**

The study found no statistically significant difference in the efficacy of neubotulinum and onabotulinum for treating forehead wrinkles, as indicated by *p*‐values above 0.05 for both static and dynamic conditions. No safety and adverse events were observed in both formulations.

**Conclusion:**

This study has demonstrated that neither formulation is inferior to each other in the treatment of forehead horizontal lines.

## 1 INTRODUCTION

Botulinum toxin (BoNT) has emerged as a versatile and pivotal therapeutic agent in modern medicine, encompassing an extensive range of clinical applications, surpassing those of many other pharmaceuticals. Originating from its early use in the treatment of strabismus and neurological movement disorders, BoNT has steadily diversified its roles over the past three decades.^1^, ^2^, ^3^ It now extends its influence into numerous medical disciplines, including ophthalmology, gastroenterology, urology, orthopaedics, dermatology, dentistry, secretory conditions, pain management, and aesthetic medicine.^4^, ^5^, ^6^, ^7^, ^8^

Within the continuously expanding realm of BoNT applications, onabotulinumtoxinA (commonly known as Botox), abobotulinumtoxinA (Dysport), incobotulinumtoxinA (Xeomin), and rimabotulinumtoxinB (Myobloc or NeuroBloc) stand as firmly established entities. Moreover, an ongoing surge of novel BoNT products is advancing through progressive stages of development.^9^, ^10^ Within the spectrum of its diverse uses, botulinum toxin A (BoNT‐A) has emerged as an invaluable tool in the realm of medical aesthetics, where it effectively addresses unwanted muscle hyperactivity.

RETRACTED

In 2002, onabotulinumtoxinA entered the United States market as the inaugural approved BoNT‐A specifically for facial aesthetic use.^11^ The approvals for BoNT‐A, including the endorsement from the United States Food and Drug Administration (FDA) for the treatment of glabellar, forehead, and lateral canthal lines, is supported by extensive research confirming both its efficacy and safety.^9^, ^12^ In some countries, such as Brazil, broader aesthetic approval allows for BoNT‐A injections across the entire face to address facial lines.^13^

The comparability of different BoNT‐A formulations, especially onabotulinumtoxinA and abobotulinumtoxinA, has been a source of contention for the past two decades. This dispute is rooted in variances such as molecular weight, excipient composition, and potency units. Ongoing conversations explore the potential impact of these distinctions on clinical efficacy and safety, with a common consensus emerging that onabotulinumtoxinA and abobotulinumtoxinA are generally considered non‐interchangeable.^14^

NeubotulinumtoxinA was developed to closely replicate the characteristics of onabotulinumtoxinA, aiming to provide a cost‐effective and easily administered alternative. It was first approved for treating blepharospasm in South Korea in 2006 and has gained substantial recognition, establishing itself as a widely accepted botulinum toxin A (BoNT‐A) product in various Asian and Latin American countries, including South Korea, Japan, Thailand, and Brazil, for both therapeutic and cosmetic applications.^14^ NeubotulinumtoxinA showed to be similar efficacy and safety profile to onabotulinumtoxinA in several different therapeutic and cosmetic applications (blepharospasm, glabellar lines, lateral canthal lines, post‐stroke upper limb spasticity, spasticity in children with cerebral palsy.^15^ Stone et al.^16^ and Kim et al.^17^ reported comparable efficacy responses between the two formulations in a murine model and it might be interchangeable based on a simple dose ratio. The aim of this study is to assess the efficacy and safety of neubotulinumtoxinA in comparison to onabotulinumtoxinA as a baseline, specifically in the treatment of forehead lines within a clinical setting.

RETRACTED

## 2 MATERIALS AND METHODS

### 2.1 Study design and patient enrollment

A 12‐week prospective, single‐blind, single‐centre, interventional split‐face study was conducted to compare the clinical efficacy and safety of onabotulinumtoxinA and neubotulinumtoxinA for forehead horizontal lines. Written consent from all subjects was obtained prior to enrollment.

### 2.2 Patient enrollment

Patients were recruited from a single centre. To qualify for study enrollment, adults needed to be between 25 and 60 years old with a desire to enhance the appearance of their forehead lines, exhibiting mild to severe severity at maximum eyebrow lift (graded on the nine‐point facial Fitzpatrick wrinkle scale). Individuals with any condition that could cause neuromuscular junction dysfunction (such as myaesthenia gravis, Lambert‐Eaton myasthenic syndrome, amyotrophic lateral sclerosis, or any systemic neuromuscular junction disorder) were excluded. Other exclusion criteria included the use of neuromuscular blocking agents, or muscle relaxants in the four weeks preceding the start of the study, previous aesthetic procedures (including botulinum toxin, filler, lasers, chemical peeling, and topical retinoid) to the forehead in the six months preceding the start of the study, individuals planning to undergo aesthetic procedures during the study, pregnant or breastfeeding participants, and those with allergies to onabotulinumtoxinA or neubotulinumtoxinA.

### 2.3 Study medication and reconstitution

Each vial of onabotulinumtoxinA and neubotulinumtoxinA contained 100U of botulinum toxin type A, 0.5 mg human serum albumin, and 0.9 mg of sodium chloride. All vials were reconstituted with 2.5 mL of 0.9% sterile, non‐preserved saline for a final dilution of 4U/0.1 mL.

### 2.4 Treatment protocol

All subjects underwent a single treatment session. Using a 34‐gauge needle, study medication was intramuscularly injected along the wrinkles. The total injection volume ranged between 4–8U for each side of the forehead; the dose per injection was 0.5U. Patients were injected with neubotulinumtoxinA to the left side of the forehead and onabotulinumtoxinA to the right side.

RETRACTED

### 2.5 Clinical outcome assessment

Prior to the injections, baseline photos at maximum lift and resting position of each subject were taken. Wrinkle scores of static and dynamic states were given by the subjects themselves and two investigators. After injections, all subjects were evaluated at 7 days, 14 days and 4, 8, and 12 weeks after treatment, both in static and dynamic states. Photographs of each patient were used for evaluation. Two investigators determined forehead line severity based on the collected photos, assessing both at maximum eyebrow lift and at rest, utilising a nine‐point scale known as the Fitzpatrick Wrinkle Scale, as outlined in a previously published study.^18^

One investigator (J. J. S.) was responsible for evaluating adverse events linked to the procedure, and participants were required to report any such events during the treatment and subsequent follow‐up appointments.

### 2.6 Statistical analysis

In this study, we aimed to compare the efficacy of neubotulinum versus onabotulinum in managing forehead wrinkles under static and dynamic conditions. The static condition (S) referred to the injection administered when the forehead muscle was not contracted, while the dynamic condition (D) pertained to injections given during muscle contraction. Participants were divided into two groups for the injection sites: the right side (R) received neubotulinum, and the left side (L) received onabotulinum.

Data were collected at baseline (week 0) and subsequently at weeks 2, 4, 8, and 12 post‐injection. To assess the treatment effect, the measurements from the five time points were summed and averaged for each condition and side. Statistical analysis was conducted using an independent t‐test to evaluate the differences between S_L versus S_R and D_L versus D_R, assuming equal variances.

## 3 RESULTS

The average summed scores for static conditions were 1.480874 (S_R) and 1.393443 (S_L), with a p‐value of 0.5472, suggesting no significant difference in the efficacy of neubotulinum and onabotulinum under static conditions. For the dynamic conditions, the average summed scores were 3.655738 (D_R) and 3.52459 (D_L), yielding a p‐value of 0.6184. Similar to the static conditions, these results indicate no significant difference between the two treatments under dynamic conditions (Figures 1 and 2). Overall, the p‐values were well above the conventional threshold of 0.05, indicating that the null hypothesis cannot be rejected for both static and dynamic comparisons. Therefore, we conclude that there is no statistically significant difference in the effectiveness of neubotulinum and onabotulinum for treating forehead wrinkles, regardless of muscle contraction status during injection.

RETRACTED

**FIGURE 1:** Before undergoing the treatment, the 32‐year‐old woman had a dynamic wrinkle score of 4. After completing the 12‐week treatment, her score decreased to 1 on both sides.

**FIGURE 2:** Prior to the treatment, the 37‐year‐old man had a dynamic wrinkle score of 5. Following the treatment, his score reduced to 2 on both sides.

### 3.1 Safety assessment

The treatment was well‐tolerated by all subjects. There was no significant difference in pain, no dizziness was reported, and swelling was not thought to be more prominent than the other side. No delayed adverse events were reported throughout the study.

## 4 DISCUSSION

Forehead lines are deemed aesthetically undesirable due to their potential to convey an aged appearance and accentuate expressions of anger, or concern.^19^ These horizontal lines emerge from the contraction of the frontalis muscle.^12^

This is the first single‐blind, single‐centre, interventional split‐face study comparing onabotulinumtoxinA and neubotulinumtoxinA in the treatment of forehead lines. These results suggest that neubotulinumtoxinA and onabotulinumtoxinA demonstrate comparable efficacy.

BoNT‐A received approval from the Food and Drug Administration in October 2017 for the treatment of forehead lines and has been studied in numerous studies since.^10^ In our study, we administered a total of 8–16 units of BoNT‐A across the entire forehead using a split‐face technique, equating to 4–8 units on each side. We employed a 1:1 dose ratio of onabotulinumtoxinA and neubotulinumtoxinA for the split‐face treatment, assuming their dosage efficacy to be equivalent because two formulations might be interchangeable based on previous murine model studies and clinical trials. Our dosage strategy deviates from the standard guideline of 20 units recommended for onabotulinumtoxinA in the treatment of forehead lines in the United States and European Union.^20^ This approach is informed by our clinical observations, as Asian individuals typically prefer more subtle and natural‐looking results. As such, we opted for a more cautious dosage approach compared to Caucasian patients, with a focus on partial rather than complete muscle paralysis to maintain facial expressiveness.

In addition to the efficacy of BoNT‐A in treating forehead lines, it is noteworthy that a study by Cavallini et al.^21^ retrospectively investigated the effect of intramuscular injection of BoNT‐A on skin texture roughness in the lateral peri‐orbital region using the Antera 3D® device. Their findings revealed a significant reduction in skin texture roughness following BoNT‐A treatment, indicating an improvement in skin texture. These results were further supported by Sun et al.^22^, who quantitatively assessed the effects of BoNT‐A treatment on dynamic wrinkles and skin quality in the upper face. Their study demonstrated a notable enhancement in pore volume, reduction of fine wrinkles, and improvement in skin texture, typically lasting from 1 to 6 months post‐injection. Collectively, these studies underscore that BoNT‐A treatment not only diminishes dynamic wrinkles but also enhances skin quality in the upper face.

RETRACTED

This study has notable limitations. Firstly, the study did not assess the duration required to return to baseline, as it did not encompass the intervals for returning to the severity of wrinkles before treatment (relapse rates). Typically, the duration of effect ranges from a minimum of three to four months, extending further with repeated injections.^23^ To comprehensively assess the longevity of the effect, studies with an extended follow‐up period are essential. Secondly, the current study did not account for individual variations in forehead contraction patterns. Despite similarities in facial anatomy, there are individual differences in muscle utilisation. Thirdly, an additional limitation of this study is its single‐blinded design. Utilising a double‐blinded approach would strengthen the study by minimising biases and providing a more rigorous evaluation of the intervention's effectiveness.

In summary, this study demonstrates that neubotulinumtoxinA administered at an equivalent dosage to onabotulinumtoxinA proved adequate in diminishing the severity of forehead lines, with a responder rate comparable to that of onabotulinumtoxinA. Noteworthy distinctions between the two study interventions were not discerned in this investigation.

## CONFLICT OF INTEREST STATEMENT

I acknowledge that I have considered the conflict of interest statement included in the “Author Guidelines.” I hereby certify that to the best of my knowledge, no aspect of my current personal or professional situation might reasonably be expected to significantly affect my views on the subject I am presenting.

## Data Availability

The data that support the findings of this study are available from the corresponding author upon reasonable request.
